# Analysis on the Policy Environment Influencing Factors of Chinese Environmental Education Development and the Reform Trend in Combination with Environmental Education History

**DOI:** 10.1155/2022/3454709

**Published:** 2022-06-21

**Authors:** Tao Yu, Manyi Gu

**Affiliations:** Southwest Medical University, School of Humanities and Management, Luzhou 646000, Sichuan, China

## Abstract

At the turn of the century, facing the challenge of information and technology, environmental education, and talent competition, the world's major environmentally, educationally developed countries have entered the wave of environmental education reform. This was promulgated in 1999, and our country also successively promulgated through “the central committee of the communist party of China under the State Council on deepening environmenta education reform and comprehensively promote quality environmental education decision” in 2001 the “basic teaching environmental education course reform outline (try out),” launched to “deepen the environmental education reform and comprehensively promote quality environmental education” for the purpose of the foundation environmental education course and teaching reform. The curriculum reform is characterized by government leadership, expert guidance, and teacher participation. Its specific approach is top-down, overall promotion, concept guidance, experimental exploration, and gradual expansion, which has achieved a lot of theoretical and practical achievements. However, the practice of more than ten years has proved that the goal of the curriculum reform of basic environmental education has not been safely realized, the classroom has not undergone fundamental changes, and the advanced curriculum concept and curriculum system have not been transformed into advanced classroom teaching practice. This paper mainly discusses the influencing factors of the policy environment of environmental education development in China and analyzes the trend of reform in combination with the history of environmental education. On the one hand, the research of this paper can enrich the research theory of pedagogy; on the other hand, it can provide reference for the practical environmental education reform and have rich significance in theory and practice.

## 1. Introduction

At the end of the last century, the United States, Britain, Germany, Japan, France, Austria, Canada, and other major environmentally, educationally developed countries as well as many developing countries carried out basic environmental education reform facing the 21st century successively or simultaneously. In 1999 and 2001, China promulgated the “Decision of the CPC Central Committee and The State Council on Deepening environmental education Reform and Comprehensively Promoting Quality-oriented Environmental education,” “Decision of The State Council on basic Environmental education Reform and Development,” and other documents to promote the curriculum reform of basic environmental education [1]. In 2001, “Basic environmental education curriculum Reform Outline (trial)” (hereinafter referred to as “outline (trial)”) was issued, marking the formal implementation of a new round of basic environmental education curriculum reform in China. The purpose of this paper is to analyze the policy environment influencing factors of environmental education development in China and the reform trend in combination with the history of environmental education, as shown in Figure 1.

## 2. State-of-the-art

### 2.1. Theoretical Significance

The curriculum has a certain degree of stability, and the teaching is alive and well. With the deepening of basic environmental education curriculum reform and the shift of focus, classroom teaching activities and teaching behavior of teachers and students will become the focus of curriculum and teaching theory and practice research.

This study clearly put forward the “three-standard” curriculum reform concept, clearly put forward to strengthen the teaching behavior research of teachers and students. It is because of the grasp of the future basic environmental education curriculum reform focus shift, so there is a certain theoretical breakthrough and innovation in the study of curriculum theory, and in some aspects, we further expand, enrich, and deepen the field and content of the study of curriculum and teaching theory, as shown in Figure 2.

### 2.2. Practical Significance

Based on summarizing the current situation and achievements of the new curriculum reform, this study examines the problems in the new curriculum reform and analyzes their attribution. Based on timely combining prudent reflection and rational evaluation, the corresponding reform strategies of basic environmental education curriculum are put forward. This not only provides corresponding theoretical guidance for the future reform of basic environmental education curriculum in China, but also has important reference value for promoting the future reform of basic environmental education curriculum [2].

Unequivocally, this study proposed “elementary environmental education curriculum reform in our country from class to class to” the study subject, then to the next step to provide a basic environmental education curriculum reform deepening of practice guidance and lead decision makers and practitioners' changing ideas of curriculum reform, that is, the true value of the classroom teaching between teachers and students, so as to play the leading and guiding role of theory to the classroom teaching practice. And we hope to play a role in changing the phenomenon of “although the course is good, the class is still the same.” This research can actually guide teachers on how to improve teaching quality in the postepidemic era, how to change their environmentally educational concepts and break through teaching ideas, which has profound practical significance.

## 3. Methodology

### 3.1. Review of Existing Studies

Throughout the relevant research of scholars at home and abroad, it is found that (1) there have been quite fruitful achievements in the subject research of “curriculum” and “classroom” at home and abroad; (2) compared with China, the research on environmental education reform theory in foreign countries is earlier, the related research content is richer, and the research is broader and deeper, especially the study on learning theory; (3) both pay attention to and advocate the application of curriculum or learning theory to classroom teaching practice. In spite of this, there are still some deficiencies in the topic research of this paper, mainly as follows:

First, there are many researches on static curriculum architecture, but few researches on concrete curriculum implementation [3]. At the beginning of the new curriculum reform, that is, since the promulgation of “Outline (Trial),” the majority of researchers and educators have to face the new “concept reconstruction movement,” which is the new curriculum idea, curriculum function, curriculum main body, curriculum objective, curriculum content, curriculum implementation, curriculum structure, curriculum evaluation, and so on: on the one hand, how the new concept is accepted by teachers and students, educators; on the other hand, it still remains in the course architecture that should be discussed.

However, there is a lack of theoretical and practical research on why the new curriculum should be implemented and how to implement it in classroom teaching.

Secondly, there are many local, superficial, and scattered researches and relatively few researches on the status of teaching activities of teachers and students in the classroom. For example, as far as the classroom teaching behavior is concerned, most literature focuses on the research of teachers' teaching behavior and students' learning behavior. However, there are relatively few researches on the “cooperation,” “interaction,” and “relationship” between teachers and students, that is, the “interaction” between teachers and students as both sides of classroom activities [4].

Thirdly, there are relatively many researches on the practice of new curriculum reform led by constructivism, postmodernism, and other foreign theories in China, but there is a lack of researches on what theories guide the specific classroom teaching practice. The debate of “what is the theoretical basis of the new curriculum reform?” and “what is the theoretical basis of the new curriculum reform?” has brought a lot of confusion to the practice of the new curriculum reform in China, which also further reflects the absence of the local curriculum and teaching reform theories in the process of the new curriculum reform.

Fourthly, in the aspect of classroom teaching practice, there are many researches using quantitative research methods, but there are relatively few qualitative researches on the classroom teaching behavior of teachers and students. Most environmentally educational researchers use questionnaires and scales to study the achievements, problems, and classroom teaching behaviors of the new curriculum reform, while qualitative research methods such as in-depth interview and observation are seldom applied, and systematic and follow-up research is also lacking [5]. It is necessary to combine quantitative and qualitative methods to grasp all aspects of the new curriculum reform.

Fifthly, there are more studies on explicit policies and measures, but less studies on curriculum reform from the perspective of culture. Although some scholars abroad such as Bruner have seen this from the angle of main body (human) development, the “cognitive” class to generate “cultural class” is the fundamental environmental education reform, and then they published the actuality of environmental education (1971), “meaningful action” (1990), “culture environmental education” (1996), and other works, to guide the reform of environmental education. However, few literatures focus on reform from the perspective of policy, system, and organizational culture, especially the internal culture of teaching practice. In the final analysis, environmental educational reform is a kind of cultural change, and the continuous renewal and development of culture are the fundamental driving forces of the new curriculum reform. We focus too much on the outward form of curriculum reform, but less attention is paid to the “daily” way of existence and the “cultural change” hidden in teaching life, such as the thinking, behavior, and value orientation of teaching subjects, principals, and environmental educational administrators. These problems are closely related to the complexity, variability, and fluidity of the whole new curriculum reform and the reality of basic environmental education in China. The solution to these problems is also complex, dynamic, and full of variables [6]. On the basis of the existing research, the study tries to grasp the achievements and problems of the new curriculum reform as a whole, focusing on the classroom, and taking the transformation of teachers and students' classroom teaching behavior, teachers' professional development, students' independent learning, school culture construction, and other aspects as the breakthrough, hoping to gain something.

### 3.2. Research on the Present Situation of New Curriculum Reform

The present study of the new curriculum reform includes two parts: one is to sort out the achievements of the new curriculum reform over the past ten years; and the other is to summarize and analyze the problems existing in the new curriculum reform. Through literature retrieval and field sampling investigation, we can grasp the great achievements of curriculum theory exploration, curriculum system construction, and curriculum text construction in the course reform of basic environmental education in the new century in more than ten years. To be specific, there exists a “curricular center tendency” that emphasizes “curriculum” over “classroom,” “teaching material” over “teacher,” and “subject” over “student.” Scheme, planning, and imagination are the root attributes of the static system curriculum. If the curriculum reform wants to bring about more profound changes and achieve the ultimate realization of all kinds of ideas of the curriculum reform, the foothold still depends on teachers to achieve and improve the classroom teaching practice as is shown in the Table 1.

### 3.3. Research on the Course Reform of Basic Environmental Education from Curriculum to Classroom

Direction research also includes two aspects: one is the direction of “where” research; the first is the study of “who.” “Where” research refers to classroom research; the study of “who” refers to the study of subjects and their behavior. The curriculum reform of basic environmental education must move from curriculum to classroom. First of all, the trend from curriculum to classroom is a response to the existing problems and reflection in the curriculum reform of basic environmental education [7]. Secondly, the direction from curriculum to classroom is the objective requirement of classroom teaching is the most basic work in environmental education. Thirdly, the trend from curriculum to classroom is the natural or necessary requirement of improving the quality of basic environmental education by classroom teaching. Fourthly, the trend from curriculum to classroom is the actual need that classroom is more important than curriculum, teachers more important than textbooks, and students more important than subjects in curriculum reform and its implementation. The fundamental trend from curriculum to classroom is to pay attention to the subject of classroom teaching and its behavior, and the key is to realize the change of the subject's behavior. Since the implementation of the new curriculum reform more than ten years ago, the phenomenon of “two skins” still exists in the reform, indicating that the teaching subject in the new curriculum reform has lost its position. The absence of teaching subject in teaching practice directly affects the improvement of classroom teaching quality. Pay attention to the growth of the subject, and let the teaching subject return; change the role of teachers, change the way of learning and communication of students, make teaching subject behavior in place, and realize the course reform from curriculum to classroom. This paper, mainly through thinking about the past, pays attention to curriculum reform and ignores the mistakes of classroom reform, summing up the experience, based on the curriculum reform from curriculum to classroom reform idea to discuss the countermeasures of realize the course reform from curriculum to classroom [8], as shown in Figure 3.

### 3.4. The Curriculum

Before the new curriculum reform, the existing curriculum structure of our country has serious deficiencies: on the one hand, school curriculum.

Secondary subject courses, subsubject courses, compulsory courses, and national courses dominate, while experience courses, comprehensive courses, elective courses, local courses, and school-based courses do not receive due attention. On the other hand, the imbalance between specific subjects in the school curriculum “has a direct impact on students' physical and mental health and overall development,” as shown in Table 2.

Take the nine-year compulsory environmental education Curriculum Plan for Full-time Primary and Junior Middle Schools (Implementation) promulgated by the State Environmental education Commission in 1992 as an example. Elementary school thought moral character, Chinese, math, social, natural, experience, music, art, labor, and other nine division and the junior middle school stage of thought politics, Chinese, mathematics, foreign languages, history, geography, physics, chemistry, biology, sports, music, art, and labor technique sorted all belong to a branch of national unified arrangement courses, compulsory courses, and subject courses, There are few comprehensive courses and elective courses [9].

In order to solve the shortcomings of the above two aspects, the new curriculum reform changes the structure of single curriculum type into a variety of curriculum type structures, so as to change the situation of extreme pursuit of subject score in teaching, low comprehensive quality of students, and poor self-learning ability, so as to promote the all-round development of students. At the same time, in order to highlight students' innovation consciousness, problem analysis, and solution ability and communication and cooperation ability, the new curriculum plan has adjusted the proportion of class hours of each discipline, so that the proportion of courses of each discipline is balanced.

## 4. Result Analysis and Discussion

### 4.1. The Influence of Environment on Environmental Educational Reform

Economic base determines superstructure: the environment will affect environmental education reform. In the wake of the COVID-19 outbreak, China has launched the world's largest “on-campus” environmental education program. In the postepidemic era, China's environmental education reform is facing a new situation based on the changes of influencing factors inside and outside environmental education, that is, the profound reform of environmental education concept, the mixed development of teaching methods, the flexible change of learning methods, the application of data in environmental education governance, and the prominent role of family environmental education [10]. At the same time, environmental education reform is facing new challenges, including the integration of online and offline environmental education, the difference between independent learning and self-management, the coordination between home environmental education and school environmental education, and the fairness of infrastructure and information literacy. To this end, the new countermeasures of environmental education reform are to use big data to serve the improvement of environmental educational governance ability, improve the ability of teachers to integrate online and offline environmental education, promote the development of personalized learning through informatization, promote the improvement of environmental education through accurate environmental educational process evaluation, and promote the efficient collaboration between home and school by using information technology as is shown in Figure 4.

### 4.2. The New Situation of Environmental Education Reform in the Post-Epidemic Era

The large-scale online environmental education practice during the COVID-19 pandemic has had a great impact on traditional school environmental education. Online environmental education has become a new normal in the development of environmental education, moving from an auxiliary form to a real, comprehensive and mainstream one [11]. The combination of online environmental education and offline environmental education has become an important form of future environmental education, which urgently requires the reform of environmental education system and the construction of a complete structured, systematic, clear, and logical environmental education system starting from environmental education practice and serving environmental education practice, as shown in Figure 5.

### 4.3. The Profound Reform of Environmental Educational Concept

The current environmental educational concept has changed from collective learning and uniformity to emphasizing individual guidance and individual learning. During the COVID-19 pandemic, “large-scale” online environmental education has become almost the only way of environmental education in China's universities and primary and secondary schools, and the entire environmental education system has taken on a major task, driving a profound change in the concept of environmental education, from class-based environmental education to a new one based on individual environmental education arrangements. In the history of environmental education development, class teaching system is the most far-reaching and still dominant environmental education and teaching method. Teachers conduct orderly environmental education for a certain number of students in specified places. Teaching activities are mainly conducted face-to-face and offline, emphasizing the concept of uniformity and collective learning [12].

Online environmental education mainly carries out environmental education and teaching with the help of environmental education technology such as network, breaks through the limitation of time and space, carries out environmental education and teaching activities, and emphasizes the idea of individual guidance and individual learning. “Internet + Environmental education” breaks through the limitation of the traditional class teaching system on environmental education and teaching at the same time and in the same space. On the one hand, a large number of course resources are put on the shelves, so that students can flexibly choose the content resources they are interested in to meet the needs of personalized development. On the other hand, high-quality curriculum resources provide strong support to weak schools and remote areas, helping promote equity and improve quality.

### 4.4. Mixed Development of Teaching Methods

The traditional teaching mode is face-to-face communication between teachers and students, while the online teaching mode is asynchronous interpersonal communication between teachers and students under the condition of time and space separation. Knowledge is no longer limited to teachers but presents the characteristics of informal, social, situational, and distributed network transmission.

Great changes have taken place in the era of teachers as the sole disseminator of knowledge. In the environmental education mainly based on the Internet, teachers need to coordinate all forces to promote the effective development of teaching activities. The hybrid teaching method, that is, the combination of the traditional classroom teaching and the current online learning of students, came into being, combining the advantages of the traditional teaching method with the advantages of the network teaching, breaking through the boundaries of teaching time and space [13]. The gradual development of mixed teaching will inevitably put forward new requirements on the teaching knowledge and ability of teachers, and the traditional role of teachers in lecturing will be transformed into the role of guiding and leading students to learn. Teachers need to update their environmental education concepts, constantly improve environmental education information literacy, guide students to adapt the environmental education reform in the Internet era, make full use of modern information technology, make teaching more rich, diversified, and personalized, and improve teaching efficiency and effectiveness.

### 4.5. Flexible Changes in Learning Styles

If environmental education is rigid and mechanical, students will be rigid and mechanical; if environmental education is flexible and adaptable, students will also be influenced by the subtle.

Traditional school environmental education usually makes strict rules and regulations for efficient management of students. Although classroom teaching gives full play to the leading and main role of teachers in teaching, it cannot give full play to students' active initiative, and the cultivation of students' innovative spirit and creative ability is still an obvious weak link. To some extent, teacher-led teaching is not conducive to the cultivation of students' creative thinking. Online environmental education prevents copying and applying offline classroom teaching methods, gives full play to the advantages of information technology, and carries out diversified student-centered learning [14].

On the one hand, online courses are not limited by time and place, and students can flexibly choose their study time according to their own time arrangement, which is recognized by students and parents. On the other hand, online environmental education to a large extent meets the needs of students to choose independently, which greatly strengthens students' autonomous learning. Students choose the content and fields they are interested in, which is conducive to realizing personalized development. Network teaching has the excellent characteristics of asynchronous interaction [15]. It can effectively conduct in-depth discussion on a topic through the network, which makes up for the defects of superficial discussion, perceptual composition, and difficulty in in-depth discussion caused by the limited time in class discussion.

Online environmental education breaks the limitation of offline environmental education time and can increase the discussion links and time. To break the way of face-to-face communication is of great help to students' full communication. Moreover, the collaborative work between groups greatly strengthens the communication between students, promotes cooperative learning, and is conducive to the development of cooperative ability as shown in Figure 6.

That is to say, the current learning style of students has improved, students are thinking and discussing more deeply, and they are communicating with each other more deeply than before. That is to say, students' learning style moves from passive to active.

### 4.6. Data Use in Environmental Educational Governance

Valet evaluation based on online environmental education carried out, including the students learning time, number, login times of discussion online homework completion, the condition of knowledge mastery, courses such as real-time evaluation, can let the teacher timely grasp the students' learning situation, dynamic adjustment, with the aid of big data, artificial intelligence technology, and personalized assessment to student's study [16].

Teachers can easily create a sequence of learning activities for a certain teaching goal through online environmental education, monitor students' learning activities at any time, judge whether students reach the standard in the learning process, and decide whether to enter the next learning activity; students can quickly enter a sequence of learning activities for efficient individual or group learning.

Through the real-time monitoring and centralized feedback of big data, as well as environmental education management departments, schools, teachers, etc. to grasp the learning situation of students in time, monitor the learning effect of students in time, and improve the way of environmental education, through centralized and timely quantitative processing of big data, subjective impression and judgment of environmental education decision makers can be avoided to a large extent, and data support can be provided for scientific environmental education governance.

That is to say, educators can use the ability of big data mining and analysis to manage students' academic performance, analyze the factors affecting students' academic performance, and analyze current teaching problems from the data level so as to make targeted improvements.

### 4.7. The Role of Family Environmental Education Is Prominent

During the COVID-19 pandemic, the impact of home environmental education has become increasingly prominent as online environmental education is carried out at home, with students shifting from “school at home” to “home schooling” and the environmental educational environment shifting from collective learning in schools to individual learning in families. Online teaching methods and family-oriented teaching scenes and teachers' environmental educational power and leading role in previous classroom teaching have been weakened and reduced, and primary and secondary school students have poor independent learning ability, weak self-control ability, unstable cognitive and psychological development, and other comprehensive factors. Parents are required to assume more important responsibilities than before in supervising and guiding students' online teaching, carrying out epidemic prevention and mental health environmental education, and communicating and interacting with teachers in home-school cooperation. Parents are even required to directly participate in home-school coenvironmental education activities to develop students' comprehensive quality and ability at home.

According to the survey, 23.4% of parents said that they always accompany their children to study online, and 29.6% said that they often accompany their children to study online. The top three things that parents help their children study online are urging and reminding their children (74.81%), downloading and uploading homework (50.54%), and logging into the learning platform (47.25%).

There are more uncontrollable factors in the learning environment at home than in school. Schools can relatively effectively control the interference factors in the campus environment and guarantee the quality of classroom teaching. However, homeschooling students face more interference, such as the attraction of entertainment platforms, the temptation of video games, and the influence of family life, which has an obvious negative impact on online environmental education. Parents play an important role in guiding and supervising online environmental education [17].

### 4.8. Integration of Online Environmental Education and Offline Environmental Education

Simply holding online teaching and temporarily replacing offline teaching substitution theory can not play the optimization of hybrid teaching.

Some teachers simply take online teaching as a simple substitute for offline teaching and carry out online teaching in traditional teaching methods, ignoring the changes of environmental educational environment and other factors, affecting the effect of online teaching. It is very important for teachers to update their teaching concepts and methods and accept and learn the ideas and technologies of online environmental education. Compared with traditional teaching, blended teaching focuses on cultivating students' innovation ability, and its teaching effect is directly reflected in students' independent learning and scientific research and creation ability. In terms of teaching methods, blended teaching emphasizes the multiple interactions between teachers and students as well as between students, and its teaching effect is directly reflected in the students' cooperation and communication ability. In terms of teaching quality, the reasonable selection and effective use of resources in hybrid teaching adapt to the needs of the development of the information society, which not only helps students expand their knowledge and expand their thinking space, but also helps students improve their ability of scientific exploration.

The effectiveness of blended teaching depends to a large extent on the teacher's attitude and ability preparation and on how the teacher makes the transition from the traditional role of face-to-face classroom to the more complex role required by blended teaching.

Some teachers are ill-prepared for online environmental education during the COVID-19 pandemic, and there have been numerous online complaints about teachers becoming anchors, teachers being unfamiliar with environmental educational software, and teachers being slow to respond. To a large extent, this reflects that the society is still unfamiliar with online environmental education, teachers' environmental educational information technology literacy needs to be improved, and students' online learning preparation is insufficient [18]. According to the survey, 7.73 percent of primary and secondary school teachers believe that online environmental education does not need to prepare lessons in advance. The top three online teaching methods of teachers are watching national or regional platform courses and teachers' centralized Q&A (56.04%), broadcasting famous teachers' courses and teachers' guidance Q&A (48.46%), and teachers' live courses (29.25%). New situation, New challenges, and New Countermeasures of China's environmental education reform in the postepidemic era 02166.8% of teachers chose “insufficient interaction.” Direct use of existing teaching resources is the main channel for online teaching methods during the COVID-19 pandemic. Online environmental education has a great impact on some subject environmental education. Online teaching of PE makes interactive information of PE teaching missing, obstacles to the creation of PE teaching situation, vacancy of PE teaching methods, and blind spots in the evaluation of PE teaching effect. Online environmental education has a negative impact on physics, chemistry, and other experimental courses that require strong operational ability. Although it has a certain promoting effect on theoretical knowledge learning, it is not conducive to the cultivation of students' practical operational ability.

Therefore, in the future teaching, the interaction between online teachers and students can be strengthened from the technical level, such as the development of VR technology and the application of 3D video technology in teaching. From the perspective of human resources, teacher training should be strengthened to improve the quality of online teaching, and the combination of online and offline teaching can be adopted.

### 4.9. The Difference between Autonomous Learning and Self-Management

With the in-depth development of “Internet + environmental education” and the in-depth promotion of online environmental education, students have more and more content and channels to learn independently. In the implementation process of online environmental education, the supervision and monitoring of environmental education itself are difficult. The independent role of students in “learning” is prominent, while the leading role of teachers in “teaching” is not enough. When students have great freedom in learning and lack necessary supervision and monitoring, it is more difficult to effectively achieve environmental educational goals [19]. In the postepidemic era, with the full restoration of normal environmental education and teaching order, it is particularly urgent to cultivate students' initiative and enthusiasm in learning and give full play to the advantages of hybrid teaching. Students' consciousness and self-discipline are important factors affecting the development and further promotion of online environmental education. Only the learners with independent and self-controlled ability can successfully complete the learning tasks in distance environmental education, and the cultivation of independent learning ability is an urgent problem to be solved.

Online environmental education is restricted by learning environment and students' independent learning ability. Teachers cannot effectively manage and supervise students' learning process, and its effect mainly depends on students' independent learning. Primary and secondary school students aged 6–18 years old, with their self-control ability being relatively weak and easy to be interfered by external factors, appear to be absent from online class. Problems such as playing games and shifting attention have a negative impact on the effect of online environmental education. The effectiveness of online environmental education largely depends on the self-control ability of students in learning, while the self-control ability of students in different regions, schools, and groups varies greatly, leading to great differences in learning effects.

Therefore, schools should find ways to improve students' learning self-control ability through teaching, so as to solve this problem.

### 4.10. Synergy between Family Environmental Education and School Environmental Education

During the COVID-19 pandemic, schools and families entered a state of collaborative environmental education, and home-school cooperation was short.

Problems gradually emerged, mainly manifested as lack of awareness and mechanism of home-school cooperation, prominent “new engineering contradiction” between parents' work and tutoring for children's learning, and inadequate matching between supervision and guidance for children's online learning at home and parents' knowledge and ability. Online environmental education at home leads to changes in school places and more opportunities for parents to be alone with their children. Parents should not only guide their children's study, but also maintain a good parent-child relationship, so the knowledge and ability of family environmental education are particularly important. However, most of the parents in China lack of preparation for family environmental education, how to carry out family environmental education, how to maintain the relationship between school and students as an important link, how to guide children's study, and growth and other issues are quite different, resulting in a huge difference in environmental educational effects.

Although problems such as out-of-school training have been eased during COVID-19, they have shifted to online training, and it is still common for parents to “value intellectual environmental education over other environmental education.” With the implementation of the policy of “suspension without suspension,” the phenomenon of some parents signing up for online training courses for their children is gradually increasing. Offline after-school training is transformed into online after-school training, which increases the academic burden of children and affects their all-round development [20]. In addition, online environmental education is mainly intellectual environmental education, while moral environmental education, physical environmental education, aesthetic environmental education, and labor environmental education encounter difficulties, and the problem of one-sided development of students becomes more and more prominent. Parents shoulder the role of educators and the responsibility of guiding children's all-round development. To help children “button their first button in life,” it is necessary to update the concept of family environmental education and improve their environmental educational ability.

Schools should actively contact and cooperate with parents and improve the coordination between family environmental education and school environmental education through parents' meeting and parents' communication of teaching philosophy.

## 5. Conclusion

This paper mainly studies the course reform of elementary environmental education in the new century from curriculum to classroom from the perspective of curriculum and teaching theory. This paper thinks that the current reform trend is the integration of online environmental education and wired environmental education, the change of teaching concept. To continue the research on this topic, the following aspects are worth pondering: (1) classroom is the center of the curriculum reform of basic environmental education, and the importance of classroom can be studied from the perspectives of sociology, ecology, management, ethics, and so on. (2) Fully explore the teaching theories guiding the future reform of basic environmental education curriculum from curriculum to classroom, especially the local excellent, traditional, or contemporary curriculum and teaching theories. After all, basic environmental education curriculum reform needs advanced, scientific, and appropriate theoretical guidance, rather than just practical operation. (3) The fundamental path of teacher professional development of the problem: teacher professional development is not only external training and training, but also teachers' self-conscious learning and independent professional development in teaching life. From the perspective of lifelong learning, teachers mainly achieve independent professional development through “internal force.” Therefore, “we must give the responsibility of professional development to teachers themselves” and let teachers carry out self-led professional development.

## Figures and Tables

**Figure 1:** Environmental educational reform matrix.

**Figure 2:** The party's overall leadership in environmental education.

**Figure 3:** Reform of the experimental teaching curriculum.

**Figure 4:** Ecological model of multiple impacts of value orientation in basic environmental education policy.

**Figure 5:** Influencing factors of teaching reform.

**Figure 6:** The proportion chart of people's different views on the changes in teaching methods.

**Table 1:** Mazmanian and Sabatier summarize the factors that influence the effective implementation of policies.

The difficulty of the question	Law control force	Illegal factors
(1) Technical difficulty	(1) Accuracy and importance of objectives	(1) Socio-economic situation and technology
(2) Differences in the behavior of target groups	(2) Compound logic of causality theory	(2) Public support
(3) Target groups as a proportion of the total population	(3) Initial allocation of financial resources	(3) Attitudes and resources of followers
(4) The extent to which a change in behavior is required	(4) Degree of integration within or between implementing agencies	(4) The support of the rulers
	(5) Decision-making rules of the implementing agency	(5) Dedication and leadership skills of executive officials
	(6) Degree of recognition of the decree by policy enforcement officials	
	(7) Official channels of contact for external personnel	

**Table 2:** Curriculum plan of nine-year compulsory environmental education full-time primary school and junior high school.

Course			Learning period grade											
			Primary school						Junior high school			Nine years		
			Week of class											
			One	Two	Three	Four	Five	Six	One	Two	Three	Total hours in primary school	Total class hours in junior high school	Total
Subject	Ideology and morality		1	1	1	1	1	1				204		404
	Ideology and politics								2	2	2		200	
	Chinese language and literature		10	10	9	8	7	7	6	6	5	1734	568	2302
	Mathematics		4	5	5	5	5	5	5	5	5	986	500	1486
	English	(I)							4	4			272	272
		(II)							4	4	4		400	400
	Sociology					2	2	2				204		608
	History								2	3	2		234	702
	Geographic									3	2		170	
	Natural science		1	1	1	1	2	2				272		
	Physics									2	3		164	
	Chemistry										3		96	
	Biology								3	2			170	
	Sports		2	2	3	3	3	3	3	3	3	544	300	844
	Music		3	3	2	2	2	2	1	1	1	476	100	576
	Arts		2	2	2	2	2	2	1	1	1	408	100	508
	Labour				1	1	1	1				136		336
	Labor technology								2	2	2		200	
	Weekly course hours		23	24	24	25	25	25	33	32	27	4964	3074	8038
	Morning meeting (evening meeting)		Ten minutes a day											

## Data Availability

The labeled data set used to support the findings of this study is available from the corresponding author upon request.
